The article "Analysis of Gait Characteristics of Patients with Knee Arthritis Based on Human Posture Estimation" was retracted in 2024. Reasons: suspected computer-generated content; unreliable results or conclusions; concerns about the data; concerns about the results or conclusions.

# Analysis of Gait Characteristics of Patients with Knee Arthritis Based on Human Posture Estimation

**DOI:** 10.1155/2022/7020804

**Published:** 2022-04-14

**Authors:** Xinyu Lv, Na Ta, Tao Chen, Jing Zhao, Haicheng Wei

**Affiliations:** ^1^School of Electrical and Information Engineering, North Minzu University, Yinchuan 750021, China; ^2^School of Information Engineering, Ningxia University, Yinchuan 750021, China

## Abstract

A gait feature analysis method based on AlphaPose human pose estimation fused with sample entropy is proposed to address complicated, high-cost, and time-consuming postoperative rehabilitation of patients with joint diseases. First, TensorRT was used to optimize the inference of AlphaPose, which consists of the target detection algorithm YOLOv3 and the pose estimation algorithm. It can speed up latency and throughput by about 2.5 times while maintaining the algorithm's accuracy. Second, the optimized human posture estimation algorithm AlphaPose_trt was used to process gait videos of healthy people and patients with knee arthritis. The joint point motion trajectories of the two groups were extracted, and the sample entropy algorithm quantified the joint trajectory signals for feature analysis. The experimental results showed significant differences in the entropy of the heel and ankle joint motion signals between healthy people and arthritic patients (*p* < 0.01), which can be used to identify patients with knee arthritis. This technique can assist doctors in determining needed postoperative joint surgery rehabilitation.

## 1. Introduction

With increases in the aging population and the accelerating pace of life, the number of people suffering from joint diseases continues to increase [1]. Orthopedic surgeons often need to use professional equipment to diagnose patients' disease conditions in diagnosis and treatment [2], but these analytical methods require specialized skills and can be painful and financially burdensome for patients [3]. In addition, it is often challenging to distinguish joint disease from gait instability, making it more difficult for doctors to judge the patient's skeletal motion state [4]. Therefore, gait analysis can determine whether there is an abnormality in a particular joint of a patient [5]. An objective determination of the patient's gait characteristics can guide clinical rehabilitation treatment [6].

Yang et al. [7] compared the gait characteristics of healthy young and aged people for dual tasks using a three-dimensional gait analysis system, which can be used as a reference for preventing falls in the elderly. Cuadrado et al. [8] proposed an extended Kalman filter (EKF) to analyze the gait of healthy subjects using optical markers and an inertial measurement unit (IMU). The results show a good correlation between the parameters obtained by the two methods. Seifert et al. [9] proposed a gait classification method based on physical features, subspace features, and harmonic modeling that correctly identified gait categories. However, the above methods have some disadvantages, such as complicated analysis processes, high cost, and long experimental cycles.

In recent years, with the maturity of deep learning technology, machine learning has gradually been applied in various areas of the medical field, such as precise cell classification [10] and image analysis for pathology [11, 12]. In addition, human pose estimation has broad application prospects in computer vision, pattern recognition, video/image sequence processing, and other technologies [13]. Cao et al. [14] developed the part affinity field (PAF) nonparametric representation method to learn how to associate body parts with individuals in an image to detect real-time multiperson two-dimensional poses. Xiu et al. [15] proposed an efficient tracker for multiperson joint pose estimation in complex unconstrained video. With the advent of times-series pose estimation algorithms, such as AlphaPose [16], human pose recognition is more convenient and faster.

Therefore, a human gait analysis algorithm based on the sample entropy fusion AlphaPose algorithm is proposed in this paper. TensorRT [17] was used to optimize the AlphaPose reasoning. Combined with sample entropy quantization, the motion trajectory signal of joint points is extracted. Statistical analysis found significant differences in the sample entropies of heel and ankle trajectory signals between patients and healthy people. This method can help doctors judge the rehabilitation of patients after operations.

### 1.1. Gait Analysis Method Based on AlphaPose Fusion Sample Entropy

#### 1.1.1. AlphaPose Human Pose Estimation

AlphaPose adopts a top-down attitude detection strategy. This method first detects the human body and then recognizes the human posture. A flowchart of the AlphaPose algorithm is shown in Figure 1.

AlphaPose consists mainly of the target detection algorithm YOLOv3 [18] and the pose estimation algorithm. First, the algorithm uses a target detection model to detect the person. After acquiring human proposals, the space transformation network (STN) adaptively transforms the input image into various spatial transformations. The spatially transformed images are then input to the single-person pose estimation (SPPE) network. The estimated human posture is then remapped to the original image coordinates using the space detransformation network (SDTN). In combination with parametric pose nonmaximum suppression (PPNMS), the pose similarity is calculated by defining the pose distance to eliminate redundant detection frames.

#### 1.1.2. Sample Entropy Algorithm

Sample entropy is widely used in gait analysis. For example, sample entropy can quantify the components of plantar pressure and torque for different activities, from sitting to walking [19]. In this paper, sample entropy is used to reflect the signal characteristics of different people's joints when they walk.

Sample entropy is a detection method to measure the complexity of a time-series signal. The higher the complexity of the signal, the larger its sample entropy. Sequences with higher self-similarity are simpler and have lower sample entropy. However, the calculation of sample entropy does not depend on the data length. The algorithmic steps for computing sample entropy are as follows:

(1) The data of *n* sample points are used to compose the time series *X*
(2) Divide the data of *n* sample points to form a time series *X*. Divide *X* into *n* − *m* + 1 arrays *X*_*m*_(*i*) of dimension *m*. *X*_*m*_(*i*) is shown in the following equation:
  (1) $$\begin{array}{c} X_{m}\left(i\right)=\left[X\left(i\right),X\left(i+1\right),\cdots ,\left(x+m-1\right)\right],\;1\leq i\leq n-m+1. \end{array}$$
 When *m* = 2, *X*_2_(*i*) = [[1, 2], [2, 3], ⋯, [*n* − 1, *n*]], 1 ≤ *i* ≤ *n* − *m* + 1. When *m* = 3*X*_3_(*i*) = [[1, 2, 3], [2, 3, 4], ⋯, [*n* − 2, *n* − 1, *n*]], 1 ≤ *i* ≤ *n* − *m* + 1. An array *X*_*j*_(*i*) of dimension *j* is compared to another vector of the same dimension. If the differences in the absolute values of their corresponding points are all less than the threshold *r*, then the two arrays are determined to be similar. If the differences in the absolute values of their corresponding points are all greater than the threshold *r*, they are not similar. Typically, *r* = (0.1–0.25) × SD, where SD is the standard deviation of the time series composed of sample point data
(3) The average probability that all vectors in the *n* − *m* + 1 arrays *X*_*m*_(*i*) of dimension *m* are similar is as shown in the following equation:
  (2) $$\begin{array}{c} \varphi_{m}=\frac{1}{N-m+1}\overset{N-m+1}{\underset{i=1}{\sum }}X_{m}\left(i\right) \end{array}$$
(4) Calculate the average probability: the dimension is increased to *m* + 1, and the above steps are repeated to obtain the sample entropy. It is shown in the following equation:
  (3) $$\begin{array}{c} SE=-\ln\frac{\varphi_{m}}{\varphi_{m+1}} \end{array}$$

#### 1.1.3. Ensemble Empirical Mode Decomposition (EEMD) Algorithm

The EEMD [20] has good adaptability in processing nonstationary nonlinear signals, and its algorithmic decomposition steps are as follows:

(1) Suppose the gait signal collected by the human posture estimation algorithm is *x*(*t*). The sequence of white noise added for *i* times is *n*_*i*_(*t*). After adding white noise, the gait signal is shown in the following equation:
  (4) $$\begin{array}{c} x_{i}\left(t\right)=x\left(t\right)+n_{i}\left(t\right). \end{array}$$
  *x*_*i*_(*t*) is the gait signal after adding white noise for the *i*^th^ time
(2) The empirical mode decomposition (EMD) [21] decomposition of the signal *x*_*i*_ after adding white noise is performed to obtain the intrinsic mode function (IMF) at different scales. It is shown in the following equation:
  (5) $$\begin{array}{c} x_{i}\left(t\right)=\overset{n}{\underset{i=1}{\sum }}C_{i,n}\left(t\right)+r_{i,n}\left(t\right), \end{array}$$
  where *n* is the number of intrinsic mode functions obtained after the decomposition of the signal *x*_*i*_(*t*), *r*_*i*,*n*_(*t*) is the residual component, and *C*(*t*) is the corresponding IMF
(3) The process of applying (4) and (5) is repeated for each addition of white noise. The *j*^th^ IMF component of *x*_*i*_(*t*) decomposed by EMD is obtained. It is shown in the following equation:
  (6) $$\begin{array}{c} x_{i,j}\left(t\right)=\overset{n}{\underset{j=1}{\sum }}C_{j,n}\left(t\right)+r_{j,n}\left(t\right) \end{array}$$
(4) The final EEMD result is obtained by averaging all the obtained IMF components as in the following equation:
  (7) $$\begin{array}{c} C_{n}\left(t\right)=\frac{1}{N}\overset{N}{\underset{k=1}{\sum }}C_{j,n}\left(t\right) \end{array}$$

### 1.2. Experiment and Analysis

#### 1.2.1. Experimental Procedure, Platform, and Subjects

The experimental procedure is shown in Figure 2. First, the human posture estimation algorithm extracts the trajectory signal of human walking joint points in the video, and this signal is normalized. The sample entropy is then calculated for the joint trajectory signal. Finally, an independent samples *t*-test is used to distinguish between healthy subjects and patients.

The experimental platform uses AlphaPose to extract the joint motion trajectories from the captured gait videos. The joint trajectory signal is uploaded to a server equipped with an Nvidia model 2080Ti GPU (graphics processing unit) for feature extraction. Finally, statistical analysis is used to distinguish between the gaits of patients with bone and joint diseases and healthy people.

An orthopedist provided the experimental data, and each test subject was informed and consented to the experiment. Twelve patients with knee arthritis were selected as the study group and 12 healthy individuals as the control group. There was no statistically significant difference between the study and control groups in general characteristics, such as gender, age, or body mass index.

#### 1.2.2. Model Acceleration of Human Pose Estimation Algorithm Based on TensorRT

TensorRT is a neural network inference engine that maximizes inference throughput and efficiency. The programmability of CUDA (Compute Unified Device Architecture) enables TensorRT to address the increasingly diverse and complex trends of deep neural networks. It is possible for TensorRT to automatically optimize the trained neural network to ensure the algorithm's accuracy and increase its speed. The accelerated reasoning process of the attitude estimation algorithm model based on TensorRT is shown in Figure 3.

In the TensorRT inference acceleration, the deep learning algorithm trained on the computer side must be transformed first. Then, the convolutional neural network of the improved model is optimized using the TensorRT analytic model, combining parameters such as precision and target deployment GPU. The optimized engine can be serialized to memory and then turned into an engine to accelerate the reasoning speed by deserialization to obtain the final prediction results. To facilitate the collection and analysis of gait videos, TensorRT is used in this paper to accelerate the processing of the human pose estimation network AlphaPose. The verification set is from MS COCO val2017 [22], and the results are shown in Table 1.

The mean average precision (mAP) of the AlphaPose_trt human pose estimation algorithm model after acceleration through TensorRT inference is 71.74%, which is unchanged compared with the mAP before acceleration. This result shows that the human pose estimation algorithm model's inferred acceleration does not affect the joint points' detection accuracy. AlphaPose_trt provides a significant improvement in inference speed and ensures human joint extraction accuracy during gait analysis. It is easy to deploy in embedded devices.

AlphaPose mainly consists of the target detection algorithm YOLOv3 and the pose estimation algorithm.  Table 2 records the inference time and the throughput of the YOLOv3 model for different batch sizes.  Table 2 shows that the batch size affects the YOLOv3 target detection model results, such as latency and throughput, which increase with increasing batch size. The inference speed of YOLOv3 based on TensorRT is faster than the original target detection model using YOLOv3 alone.  Table 3 records the inference time and the throughput of the pose estimation model for human joint point extraction for different batch sizes.

The algorithm model AlphaPose_trt optimized by TensorRT inference has lower latency, higher throughput, and faster inference speed than the original model. The results of the AlphaPose inference optimization are shown in Table 4.

When the input batch size is 1, the latency metric of the TensorRT-optimized AlphaPose_trt inference drops by 18.49 ms, while the throughput metric increases by 37.86. When the input batch size is 2, the latency indicator of AlphaPose_trt decreases by 28.18 ms, and the throughput increases by 63.86 compared to the original AlphaPose. When the input batch size is 4, the latency indicator of AlphaPose_trt drops by 37.70 ms, and the throughput increases by 97.19 compared to the original AlphaPose. These results show that AlphaPose_trt can achieve faster inference speeds without loss of accuracy.

The optimization effect of TensorRT is related to the GPU hardware performance. Batch size refers to the number of samples processed by the GPU during inference. Table 4 shows that as the batch size increases, the average latency of the processed samples decreases, and the inference time shortens. In theory, better performance hardware devices such as GPUs permit a larger batch size parameter to be set. At the same time, GPU utilization is improved when the algorithm performs inference, and the inference speed is accelerated. However, for hardware-limited devices such as the GPU, batch sizes that are too large can cause the display memory to be exceeded when the algorithm processes longer gait videos. This factor prevents the algorithm from running smoothly. After the experiments, it was found that when the batch size is four, the algorithm is the most stable for gait video inference and can significantly accelerate.

#### 1.2.3. Joint Point Extraction Based on Human Posture Estimation

The human gait video is used to extract the human skeleton and joint points through AlphaPose. The results are shown in Figure 4.

Figure 4(a) shows the gait video of some patients in the study group. Some patients with severe disease cannot walk upright and must use a walker, but walkers can easily obscure the body's joints, resulting in missed joint point detection. The complexity of the surrounding environment can also cause adverse effects. AlphaPose_trt can quickly and accurately detect human joints in the video stream, avoiding the influence of a complex environment and ensuring feature extraction accuracy for human joint trajectories, as shown in Figure 4(b). The trajectory of joint points is obtained, transformed into a one-dimensional signal, and normalized. The results are shown in Figure 5, taking the heel joint as an example.

During the video recording process, there may be complex external environmental effects such as slight lens shifts or shaking, resulting in regular upward or downward drifting of the extracted joint trajectory signal. EEMD is used to deconstruct the original signal to obtain multiple IMF components and residuals. Each IMF component is added to obtain the joint point trajectory signal with baseline drift removed for sample entropy calculation. The debaseline drift process is shown in Figure 6.

#### 1.2.4. Calculation of Sample Entropy of Joint Trajectory Signal

The extracted joint trajectory signals are characterized using sample entropy. The sample entropy is used to distinguish the joint point trajectory signal degree of confusion between the two groups and quantify the joint point trajectory signal. The study group and the control group are accurately distinguished. This method can help doctors judge the rehabilitation status of patients.

SPSS (Statistical Package for the Social Sciences) was used for the statistical analysis. An independent samples *t*-test was used to determine significant differences between the healthy and patient populations. A value of *p* < 0.05 was considered to be statistically significant. There was a difference in entropy values between the study and control groups. The entropy values of the study and control groups can be considered statistically significantly different when *p* < 0.01. The results are shown in Table 5.

In Table 5, ∗∗ indicates a significant difference (*p* < 0.01). SE_ankle_ is the ankle joint point signal sample entropy. The range of sample entropy values is 1.07±0.26 for healthy subjects and 1.49±0.27 for patients. Therefore, significant differences exist between the two groups. SE_heel_ is the sample entropy of the signal at the heel joint point, where the range is 0.76±0.20 for healthy individuals and 1.37±0.27 for patients. There were significant differences in SE_ankle_ and SE_heel_ between the two groups (*p* < 0.01).

#### 1.2.5. Analysis of Experimental Results

The patients were all suffering from joint diseases of the lower extremities, so the experiments used mainly these joints because patients' gaits would be affected by related pain or other factors. SE_ankle_ and SE_heel_ in the study and control groups were significantly different (*p* < 0.01). The main reason for this difference is that patients walk carefully to avoid accidents such as falls because of the pain in the affected area and poor balance. This behavior led to a more complex gait while walking, with more significant curve fluctuations and correspondingly larger sample entropy values. Therefore, the sample entropy values of the patient's heel and ankle signals were higher than normal.

## 2. Conclusion

Patients rehabilitating from joint surgery need professional equipment and rehabilitation judgments by doctors. The process is complicated and tedious, and the cost is high. Therefore, gait analysis through video collection has important practical significance. TensorRT has been used to optimize the inference of AlphaPose, reducing the runtime latency of the algorithm and improving its throughput. The experimental results show that TensorRT can increase latency and throughput by about 2.5 times, facilitating subsequent algorithms in embedded devices.

In this paper, the sample entropy algorithm is combined to analyze the gait of two groups of people based on human pose estimation. The algorithm quantifies the joint point trajectory signals of the study and control groups and judges whether the entropy values of the two groups' joint point trajectory signals are statistically different. The results showed significant differences in the trajectory signal sample entropies of the heel joint and ankle joint between the study and control groups (*p* < 0.01), thus distinguishing the two groups of people. Applying this method in rehabilitation judgment of joint diseases is expected to have high clinical value.

## Figures and Tables

**Figure 1:** AlphaPose algorithm.

**Figure 2:** The process of gait analysis method.

**Figure 3:** TensorRT inference optimization process.

**Figure 4:** Graph of human posture estimation results. (a) The captured human gait video. (b) The detection result of AlphaPose_trt.

**Figure 5:** Signals of heel joint point motion trajectories in both groups. (a) Patient pose estimation. (b) Patient's heel joint trajectory signal. (c) Normal pose estimation. (d) Normal heel joint trajectory signal.

**Figure 6:** The debaseline drift of heel joint point trajectory signal.

**Table 1:** Comparison of accuracy of AlphaPose before and after inference acceleration.

Method	mAP (%)
AlphaPose	71.74
AlphaPose_trt	71.74

**Table 2:** Comparison of the results of YOLOv3 inference optimization.

Mode	Batch size	Latency (ms)	Throughput
YOLOv3	1	24.49	40.83
	2	37.98	52.66
	4	53.48	74.79

YOLOv3_trt	1	13.71	72.94
	2	17.59	113.70
	4	22.96	174.22

**Table 3:** Comparison of the results of inference optimization by pose estimation.

Mode	Batch size	Latency (ms)	Throughput
Pose estimation	1	8.71	114.81
	2	8.99	222.46
	4	9.08	440.53

Pose estimation_trt	1	1.00	1000.00
	2	1.20	1666.67
	4	1.86	2150.54

**Table 4:** Comparison of results of AlphaPose inference optimization.

Mode	Batch size	Latency (ms)	Throughput
AlphaPose	1	33.20	30.12
	2	46.97	42.58
	4	62.52	63.97

AlphaPose_trt	1	14.71	67.98
	2	18.79	106.44
	4	24.82	161.16

**Table 5:** Results of the analysis of difference between the two populations.

Sample entropy	Study group	Control group
SE_ankle_	1.07±0.26	1.49±0.27^∗∗^
SE_heel_	0.76±0.20	1.37±0.27^∗∗^

## Data Availability

Data processing was supported by Ningxia Technology Innovative Team of advanced intelligent perception and control.
